The article "Computational Fluid Dynamics Analysis of Nasal Airway Changes after Treatment with C-Expander" was published in 2021. Journal: Appl Bionics Biomech.

# Computational Fluid Dynamics Analysis of Nasal Airway Changes after Treatment with C-Expander

**DOI:** 10.1155/2021/8874833

**Published:** 2021-03-31

**Authors:** Wang Xiao, Siling Liu, Yanqin Lu, Lei Lei, Ning Liu, Xiaoping Shen, Yuhong He, Ousheng Liu

**Affiliations:** ^1^Hunan Key Laboratory of Oral Health Research & Hunan 3D Printing Engineering Research Center of Oral Care & Hunan Clinical Research Center of Oral Major Diseases and Oral Health & Xiangya Stomatological Hospital & Xiangya School of Stomatology, Central South University, Changsha, 410008 Hunan, China; ^2^Xingsha Hospital, Changsha County, Hunan, No. 53 Kaiyuan Road, 410199, China

## Abstract

The use of the C-expander is an effective treatment modality for maxillary skeletal deficiencies which can cause ailments and significantly reduce life expectancy in late adolescents and young adults. However, the morphological and dynamic effects on the nasal airway have not been reported. The main goal of this study was to evaluate the nasal airway changes after the implementation of a C-expander. A sample of nine patients (8 females, 1 male, age range from 15 to 29 years) was included. The morphology parameters and nasal airway ventilation parameters of pretreatment and posttreatment were measured. All study data were normally distributed. A paired *t*-test was used to evaluate the changes before and after treatment. After expansion, the mean and standard deviation values of intercanine maxillary width (CMW) and intermolar maxillary width (MMW) increased from 35.75 ± 2.48 mm and 54.20 ± 3.17 mm to 37.87 ± 2.26 mm (*P* < 0.05) and 56.65 ± 3.10 mm (*P* < 0.05), respectively. The nasal cavity volume increased from 20320.00 ± 3468.25 mm^3^ to 23134.70 ± 3918.84 mm^3^ (*P* < 0.05). The nasal pressure drop decreased from 36.34 ± 3.99 Pa to 30.70 ± 3.17 Pa (*P* < 0.05), while the value of the maximum velocity decreased from 6.50 ± 0.31 m/s to 5.85 ± 0.37 m/s (*P* < 0.05). Nasal resistance dropped remarkably from 0.16 ± 0.14 Pa/ml/s to 0.08 ± 0.06 Pa/ml/s (*P* < 0.05). The use of C-expander can effectively broaden the area and volume of the nasal airway, having a positive effect in the reduction of nasal resistance and improvement of nasal airway ventilation. For patients suffering from maxillary width deficiency and respiratory disorders, a C-expander may be an alternative method to treat the disease.

## 1. Introduction

Maxillary transverse deficiency (MTD) is a common orthodontic problem [1, 2]. People with maxillary transverse deficiency are prone to crowded dentition, narrow upper dental arches, high palatal arches, and posterior tooth crossbites [3, 4]. This may result in a narrowed nasal cavity and cause an increase in nasal airflow resistance which may lead to a higher risk of developing obstructive sleep apnea syndrome (OSAS) [5–7]. OSAS is related to a number of systemic diseases such as myocardial infarction, arterial hypertension, and type 2 diabetes [8, 9]. Therefore, it is necessary to pay special attention to the morphology and dynamics of the upper airway, as well as maxillary transverse deficiency.

The article "Computational Fluid Dynamics Analysis of Nasal Airway Changes after Treatment with C-Expander" was published in 2021. Journal: Appl Bionics Biomech.

Rapid maxillary expansion, which is mainly used in correcting transverse maxillary deficiencies in children and adolescents, can effectively separate the midpalatal suture and broaden the nasal cavity [10]. Surgically assisted RPE (SARPE) and miniscrew-assisted RPE (MARPE) were recommended treatment methods for adult patients with transverse maxillary deficiency. However, when comparing the degree of surgical invasiveness, cost, and retention period of SARPE and MARPE, it is thought that MARPE is a more suitable treatment plan for young adults [11, 12]. A C-expander is a type of tissue bone-borne maxillary expander which consists of four miniscrews and an acrylic body. A great deal of research has verified that the C-expander, without surgical assistance, is still considered to be an effective treatment modality for maxillary skeletal deficiency in late adolescents and young adults [13–16]. However, the previous studies of the C-expander were limited to the effect of opening the midpalatal area, but the morphological and dynamic effects of C-expander on the nasal airway have not been reported.

Computational fluid dynamics (CFD) is a validated method to accurately measure and effectively compute the flow feature of the airway. This method provided us with a better way of understanding airway morphology and physiology [17–19]. CFD is also widely used in the prediction and analysis of coronary artery stenosis, myocardial infarction, salivolithiasis, and ureteral diseases, as well as several other conditions [20–23]. The growing number of CFD studies on the nasal passages has led to a better understanding of the nasal airway. Iwasaki et al. used computational fluid dynamics to analyze the changes of nasal airway ventilation after rapid maxillary expansion (RME) in a young subject, with its conclusion that RME can not only relieve nasal obstruction but also raise tongue posture in children [24]. Computed tomography scans of 4 post-EEA patients were collected and analyzed using CFD techniques. The experimental results provided a theoretical basis for CFD as a potential objective diagnostic tool for ENS [25]. Therefore, the CFD method was adopted in this study.

In all, the purpose of the retrospective study is to evaluate the nasal airway changes after the implementation of a C-expander in young adults with transverse maxillary deficiency based on the CFD method. Further detailed research is necessary to determine whether or not the use of a C-expander could significantly change the nasal airway of young adults.

The article "Computational Fluid Dynamics Analysis of Nasal Airway Changes after Treatment with C-Expander" was published in 2021. Journal: Appl Bionics Biomech.

## 2. Materials and Methods

### 2.1. Study Population

The study was approved by the Institutional Review Board of Xiangya Stomatological Hospital, Central South University (No. 20190060). Informed consent was received from the patients or their parents/legal guardians. The retrospective study includes 9 patients from the ages of 15 to 29 years (8 females, 1 male with a mean age of 18.44 ± 4.28 years), who were treated with a C-expander due to transverse maxillary deficiency from December 2015 to July 2019. All of the patients included were required to meet the following inclusion criteria:

- Greater than 15 years old
- Effective midpalatal suture expansion
- A complete set of CBCT radiographs before (T1) and within three months after expansion (T2)
- No other appliance or tooth extraction treatment during the expansion period

Exclusion criteria are listed as follows:

- Mandibular defects such as cleft lip or palate
- Failure of separation of the midpalatal suture
- Dental arch transverse maxillary deficiency

A total of nine patients were enrolled and met the inclusion criteria and exclusion criteria. Due to ethical considerations, no control group was set in this research.

The flow chart of the study is as follows: CBCT scan → model reconstruction (mimics) → mesh generation (ICEM CFD) → data acquisition (Fluent) [17, 26, 27].

### 2.2. Maxillary Expansion Design and CBCT Protocol

A C-expander is supported by four miniscrews (ORMCO TAS, America, 1.4 mm diameter, 8 mm), which were located halfway from the gingival papillae to the midpalatal suture (Figure 1). Two miniscrews were placed between the canine and first premolar on each side of the maxillary arch, and the other two were located between the second premolar and first molar. One week after the miniscrew implantation, the C-expander was bonded to the miniscrews by resin composites through four holes of it. The device was activated twice (one turn = 0.25 mm) every day until 7 mm activation was fulfilled. The gap between the anterior teeth indicates successful arch expansion. As shown in Figures 2(a) and 2(b), the arrows point to the middle palatal suture.

Patients were required to fill out the Nasal Obstruction Symptom Evaluation (NOSE) to collect information on subjective symptoms before and after expansion treatment. It includes five item scales: (1) nasal congestion or stuffiness, (2) nasal blockage or obstruction, (3) trouble breathing through the nose, (4) trouble sleeping, and (5) ability to get enough air through the nose during exercise or exertion, and scores range from 0 = not a problem, 1 = very mild problem, 2 = moderate problem, 3 = fairly bad problem, to 4 = severe problem. These numbers are summed and multiplied by 5 to give a score that ranges from 0 (no symptoms) to 100 (severe symptoms).

The article "Computational Fluid Dynamics Analysis of Nasal Airway Changes after Treatment with C-Expander" was published in 2021. Journal: Appl Bionics Biomech.

CBCT (ProMax 3D, PLANMECA Romexis, Helsinki, Finland, scan time: 8.9 s; slice thickness: 0.2 mm, 96 kV, 10 mA) images were acquired while the patient was in a natural head position with lips at rest and teeth in the intercuspal position with light occlusal contact. Patients were instructed not to swallow while the machine was being operated. The Frankfort horizontal (FH) plane was parallel to the ground, and parallel head position or a slight declination was regarded as appropriate. All CBCT images were exported as a “Digital Imaging and Communications in Medicine” (DICOM) file format.

### 2.3. Model Reconstruction

The DICOM files were read using MIMICS 21.0 (Materialism's Interactive Medical Image Control System) software, and the models were reorientated in three different planes (Figure 3). In the sagittal plane, the sagittal line was set parallel to the palatal plane. In the axial view, the sagittal line was positioned at the patient's midsagittal plane, namely, from the anterior nasal spine (ANS) to the posterior nasal spine (PNS), and the coronal line was positioned perpendicular to the sagittal line. In the coronal view, the horizontal line was tangential to the margin of the bilateral nasal floor (Figure 3). The air was segmented by setting the threshold between -1024 Hounsfield Units (HU) and -480 HU. This airway space from the nostril to the hard palate level was the area of our study. The paranasal sinuses were evacuated manually because there was almost no airflow to clear the nasal cavity. After image segmenting and region growing, the patient-specific nasal airway 3D model was obtained (Figure 4). The 3D model was then transferred to the 3-matic modeling software (Materialise), through which additional processing of the model could be completed.

### 2.4. Measurement of Nasal Airway Ventilation

After 3D reconstruction, the nasal airway geometry of STL format was loaded into ANSYS ICEM CFD (ANSYS 17.0). The nostril was created as part of the inlet, while the bottom of the nasopharynx was created as part of the outlet. Four different element sizes (A: 0.4 million, B: 1.2 million, C: 3.5 millon, D: 4.5 million) were selected to conduct a grid independence experiment. It was suggested that changes would become negligible if grid B were to be used. The maximum scale factor was set as 0.88 mm, and the max element was 0.68 mm, resulting in a computational grid of pretreatments and posttreatments consisting of 1.35 ± 0.14 million and 1.52 ± 0.15 million elements, respectively. Flow simulations were performed using the Reynolds-Averaged Navier-Stokes CFD solver (Fluent 17.0, Fluent Inc.). The air was assumed to be a Newtonian, incompressible, and homogeneous fluid. A standard atmospheric pressure (gauge pressure was 0 Pa) was set for the inlet, and a pressure of −15 Pa was applied in the outlet. The wall surface of the geometry was assumed to be stationary and a nonslip boundary. The effects of the temperature, humidity, gravity, and vibrissae factors were neglected in the simulation. To reduce the computational resources needed, steady-state condition was used in this study. The realizable *k* − *ϵ* turbulence model was selected to model the nasal airway airflow. The residual calculation was set at 10^−3^, and the iteration numbers were 1,000 steps. Second-order discretization schemes were used, and the pressure-velocity coupling was solved through the SIMPLE scheme.

The article "Computational Fluid Dynamics Analysis of Nasal Airway Changes after Treatment with C-Expander" was published in 2021. Journal: Appl Bionics Biomech.

### 2.5. Outcome Parameter

The volume (*V*) and surface area (SA) of the nasal airway morphology were quantified. The width of the midpalatal suture at the canine (MPWC) and the width of the midpalatal suture at the first molar were measured (MPWM), as well as the distances between the lateral pterygoid plates. The dental transverse measurements were made on the coronal sections of the canines, first molar, and nasal width (Figures 5(a) and 5(b)).

After simulation of the airflow, all the cross sections from the nostril to the nasopharynx were selected. The maximum pressure (*P*_max_), maximum velocity (*V*_max_), and pressure drop (Δ*P*) were measured. The nasal airway resistance (*R*) was obtained through the following formula: *R* = *R* = Δ*P*/*Q* (*Q* was nasal inlet volume flow rate). All morphology parameters and dynamic parameters are shown in Table 1.

### 2.6. Statistical Analysis

The parameters were measured two times at one-week intervals by the same researcher, and the average value was applied to the study. Intraexaminer reliability was calculated by intraclass correlation coefficient (ICC) for the measurements obtained by the examiner.

All statistical analyses were performed using the SPSS 21.0 software package (IBM, Armonk, NY). Description statistics, including the mean and the standard deviation (SD), were calculated for each variable. Normal distribution of data was tested using a Shapiro-Wilk test. For normally distributed variables, the difference between the variables before and after levels was analyzed using a paired-sampled *t*-test. For variables that were not normally distributed, the difference between the variables before and after levels was analyzed with the Wilcoxon test. Significance of the results were evaluated at the level of *P* < 0.05.

The article "Computational Fluid Dynamics Analysis of Nasal Airway Changes after Treatment with C-Expander" was published in 2021. Journal: Appl Bionics Biomech.

We performed a sample size calculation based on the difference in treatment changes of nasal airway ventilation by C-expander. To calculate the error, a power analysis using G∗power 3.1.9.2 was performed (1 − error = 0.80, *α* = 0.05, two-tailed test); the adequate sample size was 8 subjects.

## 3. Results

Intraclass correlation coefficients were greater than 0.772 for all variables in this study. No significant differences between the first and further repeated measurements were observed, which proved the reliability between the first and second measurements (ICC from 0.772 to 0.993).

As shown in Table 2, we can easily find that the average width of the nasal cavity in the treated canine area increased from 21.72 ± 1.75 mm to the 23.60 ± 1.97 mm (*P* < 0.05) measurement obtained immediately after expansion treatment. The average width of the nasal cavity in the first molar before the treatment was 29.26 ± 2.77 mm and increased to 31.52 ± 2.48 mm after the use of C-expander, and this difference was statistically significant (*P* < 0.05). The original mean distance of CMW and MMW was 35.75 ± 2.48 mm and 54.20 ± 3.17 mm, respectively. MPWC and MPWM were broadened from 0 to 2.7 ± 0.45 mm and 2.51 ± 0.46 mm, respectively.

Meanwhile, the total area and total volume were increased significantly after the use of the C-expander (*P* < 0.01 and *P* < 0.01). The nasal airway fluid dynamics results are shown below (Table 2). A pressure and velocity profile of nasal airflow is represented by one patient in our study and is shown in Figures 6(a)–6(d). It can be seen from the diagram that the changes of the velocity and pressure from the anterior nostril to the inferior nasopharynx are consistent, and the airflow pressure and velocity at the entrance of the nasal cavity are larger before and after the expansion of the arch, which indicates that the airflow pressure at the entrance is larger. The quantitative numbers of the maximum negative pressure decreased from −1.36 ± 0.60 Pa to −0.56 ± 0.46 Pa (*P* < 0.001), and the quantitative values of the maximum velocity changed from 6.50 ± 0.31 m/s to 5.85 ± 0.37 m/s (*P* < 0.001). As shown in Table 2, the values of nasal airway pressure drop reduced from 36.34 ± 3.99 Pa to 30.70 ± 3.17 Pa after the maxillary expansion treatment (*P* < 0.05). Nasal resistance was one of the most intuitive indicators of ventilation ability. In this study, nasal resistance dropped remarkably from 0.16 ± 0.14 Pa/ml/s to 0.08 ± 0.06 Pa/ml/s, and two sets of data were proven to be statistically significant (*P* < 0.05).

The article "Computational Fluid Dynamics Analysis of Nasal Airway Changes after Treatment with C-Expander" was published in 2021. Journal: Appl Bionics Biomech.

The NOSE scores showed no change after the use of C-expander, with six patients scoring from 0-0-0-0-0 to 0-0-0-0-0, and three patients scoring from 1-0-0-0-0 to 0-0-0-0-0.

## 4. Discussion

The purpose of this study was to evaluate the nasal airway changes after maxillary expansion treatment using a C-expander in young adults based on the computational fluid dynamics method. The degree of fusion of the midpalatal suture was the key element to determine the success of maxillary expansion, which is a common treatment challenge in late adolescents and young adults. Korbmacher et al. and Angelieri et al. had drawn the conclusion that chronological age was not absolutely related to the degree of fusion of the sutures in the midpalate [28, 29]. During this research, we chose a study population with a chronological age over 15 years, so that the growth potential impact could be ignored by and large. The midpalatal suture was partially or completely fused, but the structures could be clearly identified.

In this study, enrolled patients performed two CBCT scans. One was taken at the time of initial diagnosis, and the other was taken three months after the completion of the expansion. It has been proven that CBCT has low radiation dose and high accuracy [30]. Due to ethical reasons, lots of researchers took a 3-month interval to take it again [2, 31]. Research has shown that complete ossification of the midpalate suture was observed 8-9 months after rapid palatal expansion [32]. Due to this fact, we chose a time point of 3 months in this study. This time point meets the requirements of ethical concerns, as well as influence on osteogenesis.

Polysomnography (PSG) has been used as a gold standard for the diagnosis and evaluation of OSAS, which could measure respiratory indexes like apnea hypopnea index (AHI), apnea index (AI), hypopnea index (AHI), and oxygen saturation (SaO_2_) [33, 34]. Computational fluid dynamics is a verified method to compute airflow characteristic of the upper airway [17, 18, 35]. Overnight laboratory-based PSG has been used to verify the accuracy of CFD analysis of the airways and found that there was a strong correlation between negative airway pressure and AHI measures [36]. The most frequently used subjective evaluation of nasal airway function was NOSE, which is a simple and quick tool. There was little change in nasal airway function before and after expansion according to NOSE. This could be because of the self-evaluated patients who had no nasal obstruction symptoms [37, 38]. Zhao et al. [39] reported that an in vitro airway model was constructed from rapid prototyping technology, and the experimental results were very similar to CFD results. These results were further validated by the CFD simulations. After maxillary expansion treatment, the morphological changes of the nasal airway showed that the nasal cavity was broadened significantly. The hard palate is made up of two maxillary and two palatine bones, which are both closely related to the nose [40]. The midpalatal width in the canine (MPWC) was slightly wider than the midpalatal width in the molar (MPWM) in this study, and the entire palatal suture was close to parallel opening. The results were similar to Lin et al. [12] and were contrary to Zandi et al. [41]. Lin et al. inserted four miniscrews in the palate and two miniscrews in between the canines and first premolar, and the rest were situated between the second premolar and the first molar. Zandi et al.'s study used only two miniscrews to solve the problem of transverse maxillary deficiency, which produced concentrated stress and a nonparallel midpalatal suture. The main reason behind the midpalatal suture opening shape could potentially be due to the four miniscrews that were well distributed, and the stress distribution that was parallel to the midpalatal suture. We can assume that the stress distribution of four miniscrews was more homogeneous and parallel to the midpalatal suture than the two miniscrews.

The article "Computational Fluid Dynamics Analysis of Nasal Airway Changes after Treatment with C-Expander" was published in 2021. Journal: Appl Bionics Biomech.

In the present study, we applied the CFD analysis method to analyze the changes of nasal airway ventilation after the use of the C-expander. The area and volume of the nasal airway were increased significantly. At the same time, dynamic parameters like velocity and pressure in the nasal airway were decreased markedly. The relationship between morphological and dynamic trends was consistent with other studies [32, 42, 43]. A preliminary conclusion can be drawn from the previous information: that the size and shape of nasal airways can affect the nasal airflow pressure and velocity. Constricted nasal airways tend to accompany high pressure and high velocity. Once effective expansion has occurred in the nasal airway, there is a significant reduction in the pressure and velocity of the nasal airway. The nasal resistance value of the posttreatment stage was lower than that of the pretreatment stage, validating that the nasal ventilation function was improved by maxillary expansion. From the information gathered, we advise that young adults who suffer from respiratory disorders with maxillary transverse discrepancy use a C-expander to treat the disease. With the popularity of 3D printing, we can also consider this technology for the production of C-expander in the future [44].

The article "Computational Fluid Dynamics Analysis of Nasal Airway Changes after Treatment with C-Expander" was published in 2021. Journal: Appl Bionics Biomech.

There were some limits that existed within this study. Firstly, the CFD model assumed the wall of the nasal airway as hard tissue, while the nasal airway is surrounded by soft tissues, like the nasal mucosa. Secondly, the patients were awake when the CBCT machine was in operation, and therefore, an accurate image of the respiration state could not be captured. Thirdly, the posttreatment time of CBCT was delayed for three months on average, which may have led to newly formed bone deposition and bone calcification. To some extent, there was an error in measurement of the palatal suture. Lastly, there was no long-term follow-up conducted, so we could not draw a long-term conclusion about the permanent therapeutic effects of the C-expander. Therefore, we need to further evaluate the long-term efficacy and stability of the C-expander in the nasal airway in the future.

## 5. Conclusion

In the late adolescent and young adult patient, a C-expander can effectively broaden and significantly increase the area and volume of the nasal airway. This proves that the C-expander exhibited a positive effect in the reduction of nasal resistance and improvement of the nasal airway ventilation condition in the short term. For patients suffering from maxillary transverse deficiency and respiratory disorders, a C-expander may be an alternative method of treatment for the disease. The long-term impact of the C-expander on nasal airway airflow is the next step in our research.

## Figures and Tables

**Figure 1:** Four miniscrews were implanted to the maxillary.

**Figure 2:** C-expander installation: (a) before expansion; (b) after expansion.

**Figure 3:** Reorientation of CBCT sections. (a) The sagittal view shows the red line positioned through ANS and PNS which is parallel to the palatal plane, and the yellow line is perpendicular to the red line. (b) Axial view. (c) In the coronal view, the red line is tangential to the nasal floor at its most inferior level.

**Figure 4:** The region of interest of this study: the nasal airway. The upper boundary is the nostril entrance, and the lower boundary is at the level of the hard palate.

**Figure 5:** Definition of measurements: (a) measured coronal plane of the canine: intercanine nasal width (CNW), midpalatal width in the canine (MPWC), and intercanine maxillary width (CMW); (b) photographed coronal plane of the first molar: intermolar nasal width (MNW), midpalatal width in the molar (MPWM), and intermolar maxillary width (MMW).

**Figure 6:** The pressure profile of the pharyngeal airflow in (a) and (b); the velocity profile of the pharyngeal airflow in (c) and (d). (a) and (c) stand for pretreatment, (b) and (d) stand for posttreatment. ① indicates the nasal cavity; ② indicates the nasopharynx.

The article "Computational Fluid Dynamics Analysis of Nasal Airway Changes after Treatment with C-Expander" was published in 2021. Journal: Appl Bionics Biomech.

**Table 1:** Definition of measurement indexes.

Parameter	Definition
Midpalatal width in the canine (MPWC)	Distance between the left and right midpalatal sutures in the canine
Midpalatal width in the molar (MPWM)	Distance between the left and right midpalatal sutures in the first molar
Intercanine maxillary width (CMW)	Distance between the left and right cusps of the maxillary canine
Intermolar maxillary width (MMW)	Distance between the left and right maxillary bone convexities in the first molar
Intercanine nasal width (CNW)	Distance between the convexities of the right and left borders of the piriform in the canine
Intermolar nasal width (MNW)	Distance between the convexities of the right and left borders of the piriform in first molar
Total area	Surface area of the nasal airway model
Total volume	Volume of the nasal airway model
Pressure	Maximum negative pressure occurring in the nasal airway
*Δ*Pressure	Difference in value between maximum negative pressure and negative minimum pressure in the nasal airway
Velocity	Maximum velocity occurring in the nasal airway and nasopharynx
Resistance	*Q*/Δ*P* (*Q* was nasal airway inlet volume flow rate)

**Table 2:** Value of measurement indexes.

Variables	T1 (mean ± SD)	T2 (mean ± SD)	*P* value
Midpalatal width in the canine (MPWC)	0	2.7 ± 0.45	0.000^∗∗∗^
Midpalatal width in the molar (MPWM)	0	2.51 ± 0.46	0.000^∗∗∗^
Intercanine maxillary width (CMW)	35.75 ± 2.48	37.87 ± 2.26	0.000^∗∗∗^
Intermolar maxillary width (MMW)	54.20 ± 3.17	56.65 ± 3.10	0.000^∗∗∗^
Intercanine nasal width (CNW)	21.72 ± 1.75	23.60 ± 1.97	0.000^∗∗∗^
Intermolar nasal width (CNW)	29.26 ± 2.77	31.52 ± 2.48	0.000^∗∗∗^
Total area (mm^2^)	16973.53 ± 1026.03	18277.55 ± 943.35	0.000^∗∗∗^
Total volume (mm^3^)	20320.00 ± 3468.25	23134.70 ± 3918.84	0.000^∗∗∗^
Pressure_max_ (Pa)	−1.36 ± 0.60	−0.56 ± 0.46	0.001^∗∗∗^
*Δ*Pressure_max min_ (Pa)	36.34 ± 3.99	30.70 ± 3.17	0.000^∗∗∗^
Velocity_max_ (m/s)	6.50 ± 0.31	5.85 ± 0.37	0.004^∗∗^
Resistance_max_ (Pa/ml/s)	0.16 ± 0.14	0.08 ± 0.06	0.036^∗^

*M* ± *SD*: mean ± standard deviation; ^∗^*P* < 0.05, ^∗∗^*P* < 0.01, and ^∗∗∗^*P* < 0.001.

## Data Availability

The data used to support the findings of this study are available from the corresponding author upon request.
